The article "Research on the Industrial Robot Grasping Method Based on Multisensor Data Fusion and Binocular Vision" was published in 2022. Journal: Comput Intell Neurosci.

# Research on the Industrial Robot Grasping Method Based on Multisensor Data Fusion and Binocular Vision

**DOI:** 10.1155/2022/4443100

**Published:** 2022-05-25

**Authors:** Shangyu Xie

**Affiliations:** New York University Tandon School of Engineering, New York University, Brooklyn, New York, NY 11201, USA

## Abstract

At present, most of the handling industrial robots working on the production line are operated by teaching or preprogramming, which makes the flexibility of the production line poor and does not meet the flexible production requirements of the material handling system. This study proposes a solution based on adding computer binocular vision to a five-axis industrial robot system. A simple and high-precision binocular camera calibration method is proposed, the kinematics of the five-axis robot is analyzed, and the target positioning is realized; the communication between the upper and lower robots is realized through Ethernet. According to the specific target, the grasping scheme of the gripper was designed; the control software was developed using two schemes. Visual control is carried out by operating specific buttons on the control panel, and visual control is carried out by executing the macrovariable program, finally realizing the joint fusion of multisensor data and binocular vision.

## 1. Introduction

Most of the handling-type industrial robots working on production lines nowadays are operated by means of demonstration or preprogramming, which makes the production lines less flexible and cannot meet the flexible production requirements of material handling systems. As one of the most typical types of digital control equipment with a wide range of applications and high technical added value, robots are playing an increasingly important role in modern advanced production and manufacturing, and the development of robotics will be a strong driver for future production and social development [1].

While industrial robots were originally developed to free workers from the monotony of repetitive work and hazardous environments, in recent years, they have been introduced in factories and companies with the primary aim of improving productivity and quality [2].

The price of robots has fallen considerably compared to the past and will continue to fall in the future, but the cost of labour has risen worldwide and is high in individual countries and regions, which provides a wide market for industrial robots, and sales of industrial robots are growing at a fast rate [3]. There are two main applications of industrial robots in production: robotic work cells and robotic work production lines, and in foreign countries, robotic work production lines have become the main application of industrial robots [4]. The robot as the core of the automated production line to adapt to the modern manufacturing industry more varieties, less batch of flexible production development direction, has a broad market development prospects and strong vitality and has developed a variety of for the automotive, electrical machinery, and other industries of automated complete sets of equipment and production line products [5].

Robotics involves the cross-fertilisation of multiple disciplines, involving mechanics, electronics, computers, communications, control, and many other aspects. In the modern manufacturing industry, along with the expansion of industrial robots and the development of robotics, the degree of automation, intelligence, and networking of robots become higher and higher, and the functions that can be achieved are becoming more and more functional and better [6]. The connotation of robotics has changed to “an intelligent system with real action functions that flexibly applies robotics.” [7, 8]. The communication between the upper and lower robots was realized via Ethernet; the grasping scheme of the hand claw was designed for the specific target object to be grasped in the experiment; the control software was developed using both schemes. Vision control is performed by operating specific keys on the control panel, and vision control is performed by executing a macrovariable program, which finally achieves the cofusion of multisensing data and binocular vision.

## 2. Related Work

In the study by Hu et al. [9], along with the progress of science and technology and the development of production technology, the research of industrial robots based on machine vision technology has received more and more widespread attention, and a large number of scientific and technological achievements have emerged and have been well applied in actual production. A lot of work has been done on the research of industrial robots based on machine vision, and there have been many breakthrough results. The arc welding robot seam tracking control system studied by [10] uses vision sensors and image processing with neural networks to obtain seam shape data for effective seam tracking.

In the study by Li et al. [11], the XR22, a parallel robot developed by [12] incorporating a vision system for picking up parts on high-speed conveyors, can quickly pick up random goods from the conveyor and place them in order in the box by 2D positioning. The latest “second generation” picking robot from ABB of Sweden, the FlexPicker IRB360, offers the advantages of a larger payload, faster operation, and smaller footprint and with the help of simple and effective 2D vision, can quickly pick up items on a conveyor at speed of up to 2 times/second [13]. The robot vision system developed by the Finnish company RTS is successfully used in the production of naval propeller propellers, where the propeller blades are precisely ground according to CAD models by means of machine vision monitoring [14].

## 3. Introduction to the Principle of 3D Vision Measurement

In order to be able to accurately reconstruct the 3D point cloud data of the visible surface of the scattered stacked workpieces in the material frame, this study adopts binocular stereo vision plus structured light gray code [15] and phase displacement [16] for the acquisition of 3D point cloud data. The basic principle of binocular ranging [17] is shown in Figure 1, and based on the similar triangle in Figure 1, the equation can be obtained: the distances from *p* and *p*′ to the left edge of the respective imaging planes are *X*_*R*_ and *X*_*T*_, respectively, and *B* is the length of the baseline between the left and right cameras.

(1) $$\begin{array}{c} \frac{B}{Z}=\frac{\left(B+x_{t}\right)-x_{r}}{Z-f},\\ Z=\frac{B\times f}{x_{r}-x_{t}}=\frac{B\times f}{d}. \end{array}$$

In Figure 1, *O*_*R*_ and *O*_*T*_ are the main light points of the left and right cameras, respectively. If *P* is a target point to be measured in 3D space, the imaging points of *P* in the imaging planes of the two cameras are *p* and *p*′, the distances from *p* and *p*′ to the left edge of the respective imaging planes are *X*_*R*_ and *X*_*T*_, respectively, *B* is the length of the baseline between the left and right cameras, and *Z* is the distance from point *P* to the baseline, which is the spatial position of the point obtained from binocular 3D vision measurement the spatial position.

Figure 2 shows the hardware composition of the 3D vision measurement system, including two industrial cameras, a digital laser projection surface structure light projector, a six-axis robot, and a frame for storing workpieces. The process of 3D measurement of the visual surface of the workpieces in a scattered pile is to first project a number of gray code images and four phase-shift images onto the surface of the workpieces in a scattered pile using a DLP projector. At the same time, a camera is used to capture the images of the visible surface of the workpiece, as shown in Figure 3, so that the correspondence between the points (*p*, *p*′) on the left and right camera images can be determined according to the rules of gray code encoding, phase-shift, and the principle of polar line constraint of stereovision.

Based on the binocular measurement principle described in the literature [18], the 3D point cloud data of numerous workpiece surfaces in the field of view are calculated. The 3D point cloud reconstructed from the measurement of a scattered pile of workpieces is shown in Figure 4.

## 4. Target Workpiece Segmentation and 3D Matching Methods

### 4.1. 3D Matching with Model Point Cloud Generation

To determine the position of a workpiece in a loose pile, a template point cloud Ω_0_ must be obtained for 3D matching, and then, Ω_0_ must be matched in 3D with the measured and segmented 3D reconstruction point cloud Ω_*i*_ of the target workpiece in the frame to obtain the position and attitude of the target workpiece in the loose pile in the frame.

There are two ways to obtain a 3D matching template point cloud of a workpiece.  Figure 5 shows a CAD theoretical model of the workpiece obtained from the production unit, which is discretely processed to obtain a point cloud of the entire external surface of the workpiece.  Figure 6 shows a template point cloud formed by measuring, reconstructing, and stitching a single workpiece in situ using the 3D measurement system developed in this study. Although the template point cloud Ω_0_ generated by the CAD model has better detail, the method of obtaining the template 3D point cloud Ω_0_ by in situ measurement has the advantage of being simple to use and easy to operate. This study shows that the accuracy and effectiveness of the two methods in 3D matching are basically the same.

### 4.2. Target Workpiece Segmentation Algorithm

There is no good method for segmenting the target workpiece from a 3D point cloud of a scattered pile of workpieces. Considering that this measurement system uses binocular vision and reconstruction through multiple sequential images and that the projecto's light projection pattern is controllable, it is possible to obtain a 2D image of the workpiece in a scattered pile by projecting a uniform, intensity-controlled illumination source. The two-dimensional image is then divided into different regions by segmentation of this two-dimensional image; then, the three-dimensional point clouds corresponding to the two-dimensional image regions are also divided differently in the three-dimensional scene, so that the three-dimensional point cloud data subsets belonging to different individual workpieces can be roughly distinguished. Segmenting the scattered workpieces in the material frame from the 2D image is a feasible way to reduce the complexity of 3D spatial segmentation algorithms and improve the efficiency of 3D matching.

Common 2D image segmentation algorithms include the binarisation method, watershed method [19], and edge method [20].  Figure 6 shows the results of the test image segmentation process using the edge method. In this study, this method is used to segment the scattered piles of workpieces in the material frame on 2D images to initially identify the target workpieces and the 3D point cloud subsets to which they belong.

### 4.3. Three-Dimensional Matching Algorithm

When using ICP algorithms, it is often necessary to use the PCA (principal component analysis) method in order to obtain a good initial pose and thus improve the speed and accuracy of ICP alignment.

As shown in Figure 7, if the point cloud consists of *m* points, let *X* be a 3 × *m* matrix containing the coordinates of all the points; the coordinates of the centre of gravity of the point cloud are *μ*. First, the point cloud is translated, and the origin of the new coordinate system is the centre of gravity of the point cloud *μ*. The new 3 × *m* matrix of the point cloud is obtained after the translation transformation *X*_*μ*_. By constructing the covariance matrix cov *X* and obtaining the eigenvectors corresponding to the largest eigenvalues of cov *X*, we further construct the rotation transformation matrix *R*, which is orthogonal and satisfies the right-hand system rule; using the rotation transformation *R* to rotate *X*_*μ*_, we obtain **X**_out_.

(2) $$\begin{array}{c} X_{\mu }=X-\mu ,\\ \mathrm{cov}X\;=X_{\mu }\times X_{\mu }^{T},\\ X_{\text{out}}=R\times X_{\mu }. \end{array}$$

The template point cloud Ω_0_ and target point cloud Ω_1_ are both transformed by PCA (at this point, the template point cloud Ω_0_ and the target point cloud Ω_1_ are both described in their respective centre of gravity coordinate systems) and then further matched by ICP to obtain the final 3D point cloud positional matching results.

(1) The nearest distance principle is used to obtain the relationship between the template point set *M* = {*q*_*i*_} (*i* = 1, 2, 3,…, *L*) and the corresponding points in the target point set *S* = {*p*_*j*_} (*j* = 1, 2, 3,…, *K*) to obtain the set of one-to-one pairs of points {(*q*_1_, *p*_1_)(*q*_2_, *p*_2_); …; (*q*_*i*_, *p*_*i*_) …; (*q*_*N*_, *p*_*N*_)}. is the set of target points *S*, “∗” is the set of template points *M*, and the connecting line indicates the pairing relationship between the points. *R* and *T* are the rotational and translational transformation matrices between the target and model point sets as shown in Figure 8.
(2) Find the new positions of the model point set *M* and the target point set *S*, respectively, after the centre of gravity coordinates *C*_*S*_, *C*_*M*_, and *p*_*i*_ of the point cloud has been transformed by the *R* matrix to *ρ*_*i*_′; let the average pairwise distance in the transformed matching by ICP be *E*; the purpose of the ICP iteration is to find *R*, such that *E* is minimized.
  (3) $$\begin{array}{c} C_{S}=\frac{1}{N}\sum_{i=1}^{N}p_{i},\\ C_{M}=\frac{1}{N}\sum_{i=1}^{N}q_{i},\\ \rho_{i}^{\prime }=C_{M}+R\left(p_{i}-C_{s}\right),\\ E=\frac{1}{N}\sum_{i=1}^{N}{\left\|q_{i}-\rho_{i}^{\prime }\right\|}^{2}. \end{array}$$

## 5. Experimental Results and Analysis

The object of this test is a white packaging bottle as shown in Figure 9. The two-dimensional image of this target object has good edge characteristics. The image was first acquired by the left camera in the binocular vision system and edge segmented to be able to distinguish and label individual individuals. The result of edge processing of the image is shown in Figure 10.

After edge processing, the image often has broken edges as shown in Figure 9, which is detrimental to the segmentation of objects using the connected-domain method and must be effectively edge repaired.

Figure 9 shows the partial edge fracture after Canny treatment and partial fracture repair.

The approach used in this study is as follows: for edge images, a Gaussian template is used for filtering and a Gaussian value is calculated for the white pixels close to the black pixels, resulting in reduction in the gray value of the white pixels. The Gaussian template is applied to the edge image and then binarised, increasing the width of the edge lines and effectively filling in the local breaks caused by the edge operator calculation.

## 6. Conclusions

A binocular 3D measurement system based on gray code structured light and phase-shift structured light was established by improving the robot to reconstruct the scene of scattering workpieces. In order to correctly segment the scattered parts and match the 3D pose of the target workpiece, this study first uses the edge features of the scattered parts to segment the 2D image to obtain the image area of the target workpiece and then uses the principle of optical geometric imaging to take the segmented 2D image as in segmenting a 3D point cloud. The three-dimensional visual inspection results of the parts are used to control the six-axis robot to grab the parts, and the effect is good. It is very helpful to our future production, greatly shortens the working hours, and reduces the cost of the enterprise.

## Figures and Tables

**Figure 1:** Principle of binocular distance measurement.

**Figure 2:** Hardware components of the 3D measuring and sorting system.

**Figure 3:** Image formed by a line structured light projected using gray's encoding technique. (a) Left camera image. (b) Right camera image.

**Figure 4:** Reconstructed 3D point cloud scene in a scattered pile state.

**Figure 5:** Workpiece field measurement to create a model point cloud Ω_0_. (a) Correct correspondences. (b) Faulty correspondences.

**Figure 6:** Image edge processing. (a) Original image. (b) Edge processing image.

**Figure 7:** Test point cloud data for PCA transformation.

**Figure 8:** Pairing the target point set with the template point set using the nearest distance principle.

**Figure 9:** Connected domains and area filtering.

**Figure 10:** Edge segmentation processing.

## Data Availability

The datasets used to support this study are available from the corresponding author upon request.
